RETRACTED

# Study on Damage Mechanism and Repair of Vascular Endothelial Cells Based on Ultrasound Technology

**DOI:** 10.1155/2021/6680356

**Published:** 2021-03-13

**Authors:** Shuhao Deng, Quan Jiang, Xin Lu, Yuan Zhang

**Affiliations:** ^1^Department of Ultrasound, Pudong New Area People's Hospital Affiliated to Shanghai University of Medicine & Health Sciences, Shanghai 201299, China; ^2^Department of Radiology, Pudong New Area People's Hospital Affiliated to Shanghai University of Medicine & Health Sciences, Shanghai 201299, China; ^3^Department of Ultrasound, Pudong New Area People's Hospital Affiliated to Shanghai University of Medicine & Health Sciences, 490 Chuanhuan South Road, Pudong New Area, Shanghai, China

## Abstract

**Objective:**

To detect the endothelial function of external iliac artery in rats with different stages of atherosclerosis by high-resolution ultrasound, so as to provide experimental methodological basis for evaluating the function of vascular endothelial cells by ultrasound.

**Methods:**

The animals were randomly divided into the control group (*n* = 6) and the atherosclerosis model group (*n* = 15). The atherosclerosis group was further divided into 4-week group, 8-week group, and 12-week group, with 5 animals in each group. After separating and grinding rat spleen, the obtained cells were cultured by density gradient centrifugation. After the cells adhered, the morphology of the cells was observed under a microscope and identified by DiI-Ac-LDL and FITC-UEA-I double staining. The activities of LDH and SOD, the contents of MDA and GSH, and the contents of NO in plasma were detected by biochemical methods.

**Results:**

The protective effect of rosanilin on brain injury in rats with acute hypobaric hypoxia and its regulation on the expression of pAkt protein; ox-LDL inhibited the proliferation activity of EPCs in a concentration-dependent manner. The expression of KLF2 and S1PR1 in HAEC can be knocked down by small interfering RNA, and knocking down KLF2 can not only downregulate the expression of S1PR1 but also downregulate HAVEN. With the development of atherosclerosis, the endothelium-dependent relaxation function and endothelium-independent relaxation function of the control group and the atherosclerosis model at 4, 8, and 12 weeks were damaged in different degrees and gradually aggravated.

**Conclusion:**

Atherosclerosis is a disease with both morphological and functional damage, and vascular endothelial function is damaged in the early stage with corresponding pathological changes. Ultrasound is an effective method to evaluate vascular endothelial function.

## 1. Introduction

Vascular endothelial cells not only have physiological barrier function but also have extremely active metabolic function. Patients with coronary heart disease are often accompanied by endothelium-dependent dilation disorder of brachial artery and coronary artery, which suggests that these two sites are interrelated and that endothelial dysfunction is a systematic disease in atherosclerosis. Many factors can induce the formation and development of atherosclerosis. Therefore, exploring the factors and mechanism of vascular endothelial cell injury has become the focus of cardiovascular research.

RETRACTED

Nowadays, ultrasound technology has been widely used to evaluate vascular endothelial function. At present, the methods used are mainly based on the diastolic dysfunction caused by endothelial cell injury. Ultrasonic cavitation can damage the vessel wall, increase the permeability of the vessel wall, shed endothelial cells, rupture and bleed the vessel wall, and form thrombus and other biological effects, which have been confirmed in the study of rat ear vein, myocardium, mesentery, spleen microvessels, and various tumor tissue microvessels [1]. When vascular endothelium is damaged, active substances change, vasoconstriction spasm, platelet self-coagulation, smooth muscle cell proliferation, and vascular remodeling, that is, vascular endothelial dysfunction. At the same time, it can activate platelets, promote monocyte adhesion and thrombosis, produce inflammatory reaction, and affect lipoprotein metabolism, uptake, and blood vessel growth and remodeling [2]. Acoustic contrast agents have unique application value in this field. It is possible to find microscopic lesions from macroscopic imaging by using the interaction of microbubbles with endothelial cells and leukocytes and their backscattering characteristics.

Vascular endothelium has many regulating functions. At present, the function of vascular endothelium is often evaluated by the response of blood vessels to drugs or mechanical stimulation. In this paper, the endothelial function of the left external iliac artery of rats in different stages of atherosclerosis was detected in vivo by high-resolution ultrasound, and related pathological examination was carried out, in order to provide morphological basis for the method of evaluating the function of vascular endothelial cells by peripheral artery ultrasound.

## 2. Related Work

Mittal et al. [3] think that besides the cavitation effect caused by ultrasonic irradiation of microbubbles, it can damage microvessels, and the possible reasons include that cavitation effect can promote the absorption of paclitaxel by tumor tissues, promote the apoptosis of tumor cells, and reduce the secretion of angiogenic factors such as VEGF, thus reducing angiogenesis. Shosha et al. [4] specifically deleted cardiac ATG5, which led to the early expression of aging phenotype, and began to die from six months of mice. Compared with wild-type mice, mice without ATG5 showed myocardial hypertrophy, fibrosis, and abnormal mitochondria in old age [5]. Fittipaldi et al. [6] found that miR-30a can negatively regulate autophagy in tumor cells. Since then, a large number of studies on the influence of noncoding RNA on autophagy have begun. Manetti et al. [7] found that the increase of miR-144 levels in myocardial cells and circulation during ischemic preconditioning may be helpful to maintain the level of miR-144 during ischemia reperfusion. miR-144 binds to mTOR in a targeted manner, thus activating autophagy, improving myocardial function, and reducing infarct size. The inhibitor of miR-144 can weaken the protective effect of preconditioning on reperfusion injury. This suggests that the protective effect of preconditioning may be partly realized by autophagy regulated by microRNA.

RETRACTED

Xing et al. [8] compared the endothelium-dependent vasodilation function of healthy people after blocking the upper arm or forearm and found that blocking the brachial artery dilatation of the upper arm is more obvious, which may be due to the brachial artery ischemia caused by blocking the upper arm. Zhao et al. [9], with combined PEI therapy, found that the ablation volume of the liver was significantly increased, which was 10 times larger than that of PEI alone. In Eloueyk et al.'s study [10], nonnitrate vasoactive drugs have no obvious effect on brachial artery reactivity, so these drugs can be used continuously before the test. Research by Xuan et al. [11] shows that blood flow acting on G protein on endothelial cells can trigger various phosphorylation processes in endothelial cells, which leads to rearrangement of vascular endothelial cells along the blood flow direction and at the same time regulates signal transduction pathway mediated by nuclear factor kB, thereby regulating the expression of various genes in endothelial cells, resulting in changes in the structure and function of blood vessels.

## 3. Materials and Methods

### 3.1. Material

Twenty-one experimental rats, aged 3.0-5.0 months, weighing 1.65-2.15 kg, of either sex, were fed in a single cage, drinking water freely, feeding at 20.3°C, and given regular illumination (12 hours each day and night).

### 3.2. Experimental Method

#### 3.2.1. Culture of Spleen-Derived EPC

The spleen of rats was isolated and grinded in sterile environment, washed with PBS, and filtered with 200 molybdenum sieve to obtain the mixed solution of spleen cells. The oxygen cabin was controlled by a computer to reach the atmospheric pressure at an altitude of 7000 m within 15 min, simulating acute hypobaric hypoxia for 18 h (temperature 15 ± 2°C, humidity 30% ± 5%). Within 15 minutes after the end of hypoxia, the pressure in the low-pressure oxygen chamber was reduced to the atmospheric pressure at an altitude of 150 m (the altitude in the experimental area). The cells were inoculated into a 24-well cell culture plate at a cell density of 10^4^/well. After the cells were completely fused, scratches were made with a 200 *μ*l gun head. When the melting ratio reached 70%, the frozen tube was taken out, the outer wall of the frozen tube was sterilized with 70% alcohol, and the next operation was carried out on the ultraclean workbench. Blood was collected from the abdominal aorta, anticoagulated with heparin, centrifuged at 3500 rpm/min for 10 min, and the upper plasma samples were collected. The NO content in the blood of rats in each group was detected and calculated according to the following operation steps.

RETRACTED

#### 3.2.2. Establishment of Animal Model

The animals were randomly divided into the control group (*n* = 6) and the atherosclerosis model group (*n* = 15). The atherosclerosis group was further divided into 4-week group, 8-week group, and 12-week group, with 5 animals in each group. The animals were fed adaptively for one week, and then, the control group was fed with ordinary pellet feed. In the atherosclerosis group, 2 g cholesterol mixed with a little common pellet feed was fed first every day, and normal pellet feed was given after it was eaten up, with a daily feed amount of about 150 g.

#### 3.2.3. Tissue RNA Extraction

Tissue grinding: prepare liquid nitrogen tank, high-pressure scissors, and tweezers; add 1 ml TRIzol to a magna tube; on the ice box, when the tissue becomes soft, cut off 100 mg of tissue, fully cut it into pieces in magna tube, and quickly throw the rest into liquid nitrogen; in the homogenizer, the speed is 6500 rpm for 15 s, and the cooling time is 10 s on the ice tray, which is repeated 3-5 times; save at -80°C.

RNA extraction: 0.5 ml TRIzol/hole (1 ml TRIzol/l00 mg tissue), take it out from -80°C refrigerator and melt it at room temperature; 0.1 ml chloroform, vortex l5 s, standing at room temperature for 5 min; according to the measured standard curve, the measured OD45O value was converted into the number of viable cells, and the inhibition rate of sodium arsenite on cell proliferation was calculated. According to the size of glue, cut PVDF membrane with corresponding size, mark it, and soak it in methanol solution for 10-15 seconds. 10% homogenate was prepared, centrifuged at 3000 rpm/min for 10 min, the supernatant was sucked, and the contents of MDA and GSH and the activities of LDH and SOD in brain tissue of rats in each group were detected and calculated according to the following operation steps.

RETRACTED

#### 3.2.4. HE Staining

After the rats in each group were decapitated, the right hemisphere was fixed with 4% paraformaldehyde, dehydrated with gradient ethanol solution, transparent with xylene, embedded in paraffin, and sectioned continuously. Paraffin sections were dewaxed with xylene, dehydrated with gradient alcohol, and soaked in distilled water for 1 min. Stain with hematoxylin for 10 min and wash with deionized water for 1 min × 2 times; differentiation with 1% dilute hydrochloric acid alcohol solution for 20 s, deionized water washing for 1 min × 2 times; blue the nucleus with 1% weak ammonia water for 1 min, and wash it with deionized water for 1 min × 2 times; dye with eosin for 10 min and soak in deionized water for 30 s, sequentially dehydrating with 70%, 80%, and 90% ethanol once and dehydrating with 95% ethanol and 100% ethanol twice, each time for 1 min; xylene is transparent for 1 min × 3 times. The pathological changes of brain tissue of rats in each group were observed under the microscope.

### 3.3. Statistical Treatment

All the data are expressed by means of mean standard deviation, and SPSS 19.0 is used to process the data conforming to normal distribution by *t*-test (comparison between two groups) or one-way analysis of variance (comparison between multiple groups). *P* < 0.05 is a significant difference.

## 4. Result

### 4.1. EPC Culture and Identification

#### 4.1.1. Morphological Characteristics of EPC

The EPCs (endothelial progenitor cells) successfully isolated and cultured were observed under an inverted phase contrast microscope, as shown in Figures 1(a) and 1(b); the cells were evenly distributed in a circle on the first and second days of culture. On the third day of culture, as shown in Figure 1(c), most of the cells adhered to the wall, and some cells showed small protrusions. On the 7th day of culture, as shown in Figure 1(d), the cultured cells grew and increased, and the cells extended like spindle, showing typical EPC morphology.

#### 4.1.2. Effect of ox-LDL on Proliferation of EPCs

The EPCs were treated with ox-LDL with different concentrations (0 *μ*g/ml, 10 *μ*g/ml, 30 *μ*g/ml, 60 *μ*g/ml, and 100 *μ*g/ml). By RTCA test, we found that the proliferation curve was basically at the same baseline level before adding ox-LDL. After adding different concentrations of ox-LDL to treat EPCs, the cell proliferation curve was significantly different. With the increase of ox-LDL concentration, the proliferation activity of EPCs also increased. The proliferation curve obtained is shown in Figure 2.

RETRACTED

#### 4.1.3. Under Normal Environment, the Influence of Autophagy Level on the Proliferation Ability of EPCs

To test the effect of autophagy on EPC proliferation, we used shAtg7 lentivirus to inhibit autophagy-related gene ATG7, thus inhibiting autophagy. After lentivirus shAtg7 was transfected, we detected the proliferation activity of EPCs by RTCA. We found that the proliferation curve of shATG7 alone did not change significantly compared with control, as shown in Figure 3. This indicates that autophagy itself does not affect the proliferation ability of EPCs in normal environment.

### 4.2. Biochemical Index Test Results

#### 4.2.1. Detection Results of NO Content in Plasma

Compared with the control group, the NO content in plasma of rats in the atherosclerosis model group decreased significantly (*P* < 0.05). Compared with the hypoxia model group, the content of NO in plasma of rats in high- and low-dose groups of *Rosa multiflora* and dexamethasone group increased significantly (*P* < 0.01 or *P* < 0.05) (Figure 4).

#### 4.2.2. Results of Brain Water Content Measurement

Compared with the control group, the brain water content in the atherosclerosis model group increased significantly (*P* < 0.01). Compared with the hypoxia model group, the brain water content of rats in the high- and low-dose groups and dexamethasone group decreased significantly (*P* < 0.01 or *P* < 0.05) (Figure 5).

#### 4.2.3. Histopathological Changes

The results of HE staining showed that the pia mater and cerebral cortex of rats in the normoxic control group were closely attached, and red-stained red blood cells were rarely or not seen. The cerebral cortex is uniformly red-stained, the cells are evenly dispersed, round or polygonal, the nucleus is blue-stained, the cytoplasm is red-stained, and the spaces around the capillaries are uniform. The pyramidal cells in the hippocampal area were arranged in order and uniform in size, with blue light-stained nuclei and red light-stained cytoplasm (Figure 6). After 18 hours of acute hypobaric hypoxia, there was obvious separation between the pia mater and the cerebral cortex, and a large number of red-stained red blood cells could be seen in the gap. Hematoma with deep red staining can be clearly seen in the cerebral cortex, most cells are deeply stained with blue, showing obvious shrinkage and deformation, a few cells are swollen and lightly stained, and capillaries become thicker and the surrounding space becomes larger.

### 4.3. HAEC Is Regulated by Transcription Factor KLF2

To investigate whether HAEC (human aortic endothelial cells) is involved in the KLF2 and S1PR1 pathways, we constructed siRNA of S1PR1 and KLF2. Because the effect of a single small interfering RNA transfection is less than 6 days, we conducted two siRNA transfection with the same amount in the first 12 hours of NG culture. QRT PCR was used to detect the mRNA expression level. The results showed that siRNA knockdown S1PR1 and KLF2 in HAEC, respectively, and knockdown S1PR1 did not change the expression of HAVEN (Figure 7(a)); KLF2 knockdown not only downregulated the expression of S1PR1 but also downregulated the expression of HAVEN (Figure 7(b)).

RETRACTED

Therefore, we suspect that HAVEN, KLF2, and S1PR1 can regulate each other and regulate vcam-1 and Enos systems downstream of them. There is a close interaction between HAVEN-KLF2-S1PR1, but the specific regulatory mechanism of HAVEN in regulating endothelial cell injury induced by hyperglycemia needs further study.

### 4.4. Endothelium-Dependent Relaxation Function and Endothelium-Independent Relaxation Function of External Iliac Artery of Rats in Each Group

Under a light microscope, no evidence of atherosclerosis was found in the external iliac artery of the normal control group and the 4-week atherosclerosis model group. The endothelial cells were continuous and complete, the internal elastic membrane structure was clear, the tube wall thickness was uniform, and the cells were arranged orderly. In the 12-week group of atherosclerosis model, under a light microscope, the morphology of endothelial cells was irregular and discontinuous, the inner elastic membrane was interrupted, smooth muscle cells proliferated to the intima, and plaques were seen protruding into the lumen. Under an electron microscope, endothelial cells in the normal control group were flat (Table 1).

## 5. Discussion

The imbalance between vascular homeostasis and remodeling is the core pathogenesis of many chronic vascular diseases. Among them, the abnormal function and structure of vascular endothelial cells are an important initial link, which is a typical manifestation of the imbalance between vascular homeostasis and remodeling in atherosclerosis. Recurrence after endovascular embolization refers to recanalization of tumor body or neck after complete embolization and residual neck and cavity enlargement after partial embolization. Guanghao et al. [12] found that high glucose level can increase the expression of MALAT1 and confirmed that MALAT1 can upregulate glucose-induced inflammatory mediators TNF-*α* and IL-6 by activating amyloid antigen 3. Some scholars used low-pressure oxygen chamber to simulate different altitudes, established rat brain hypoxia injury model, and observed the brain edema of rats with different degrees of hypoxia. The results showed that low-pressure hypoxia can induce brain edema in rats, and the degree of brain edema in rats increased with the increase of hypoxia height [13, 14].

RETRACTED

Studies have shown that MALAT1 can regulate gene variable shearing by regulating phosphorylation of SR shearing factor [15]. Hai-Bo et al. [5] found that MALAT1 silence significantly inhibited the proliferation and migration of human osteosarcoma cells and speculated that PI3K/AKT signal played a certain role in promoting it. Xiao et al. [16] think that the recurrence after operation is closely related to the size of intracranial aneurysms, and the recurrence rates of aneurysms smaller than 10 mm and larger than 10 mm are 16.9% and 36.0%, respectively. Aziz et al. [17] used a self-developed small pulse focused ultrasonic cavitation therapeutic instrument combined with lipid microbubbles to block the microcirculation of vx2 subcutaneous tumor in rats and found that the grayscale value of tumor radiography decreased from 67.8 ± 13.3 before treatment to 29.7 ± 20.1, and there was no obvious recanalization after more than 60 min. Under a light microscope, the tumor microvessels were slightly dilated and congested. However, other studies have shown that there is no significant difference between FMD measured by blocking forearm and upper arm of subjects with or without cardiovascular risk factors, that is, it is feasible and accurate to measure FMD by blocking the upper arm or forearm [18].

Clinically, the function of vascular endothelium is often evaluated according to the change of blood vessel inner diameter [19]. Invasive methods, such as angiography and intravascular ultrasound, have been used to measure endothelial function in the early stage, but they are expensive and increase patients' pain, so they are not easy to popularize and cannot be repeated and observed dynamically. He [20] measured the change of inner diameter of peripheral artery before and after congestion in 40 healthy people with the same instrument. The result showed that the total coefficient of variation of endothelium-dependent vasodilation was 1.8 (female 1.6, male 1.9%, *P* = 0.18). It has been found that vein transplantation of endothelial progenitor cells into mice with carotid artery endothelial injury can promote the reendothelialization of injured artery and reduce neointimal hyperplasia. Because the expression of endothelial cell adhesion molecule in normal vascular endothelial cells is very little and when the endothelial function is damaged the expression is significantly increased, an acoustic contrast agent with endothelial cell adhesion molecule ligand on the surface can be designed to target the lesion site and combine with damaged endothelial cells. Therefore, finding new lncRNA in diabetic secondary vascular diseases, studying its molecular regulation mechanism, and exploring its application in clinical diagnosis and treatment are the new direction and new hot spot of translational medicine research on diabetic cardiovascular diseases and also the biggest feature of this study.

RETRACTED

Clinically, an easy-to-understand way is needed to fully understand and evaluate the risk of postoperative recurrence. However, it is extremely difficult to predict the rupture of arterial hemangioma, and its success rate is about 2% per year [21]. However, p-AKT/AKT has been widely used in the research of related pathway molecules of cell proliferation. SC-79 was used as an agonist of PI3K/AKT/mTOR PTEN-Akt and other pathways in bladder epithelial cancer cells, human glioblastoma cells, human gastric cancer cells, and pancreatic ductal cancer cells [22, 23]. The upregulation of AQP1 level in brain tissue is closely related to the occurrence of brain edema. Weisheng et al. [24] showed that inhibiting AQP4 expression can alleviate brain edema caused by ischemic brain injury. This is inconsistent with the discovery by Li et al. [25] that the WNT/Ca^2+^ pathway and MALAT1 can be activated simultaneously in gliomas. However, Raymond classification has some limitations and subjectivity. Because the recurrence of aneurysm after operation is affected by many factors and there is a large difference in embolic density in the same classification, the accuracy judgment and application of Raymond classification in clinic are limited to a certain extent [26]. Among them, HAVEN is the focus of this study. For the first time, the specific mechanism of HAVEN regulating the inflammatory response of vascular endothelial cells induced by high glucose was studied to clarify the upstream and downstream regulatory pathway of S1PR1-mediated endothelial cell changes stimulated by high glucose and the role of HAVEN in it.

Pulsed HIFU with low duty cycle can also achieve high peak negative pressure, so some scholars speculate that it can also produce similar vascular endothelial cell damage, which avoids the thermal effect of HIFU with high duty cycle. Studies from different angles suggest that blocking the upper arm will also cause brachial artery collapse, and it is more difficult to obtain satisfactory images, which will lead to the loss of image information. Blocking the forearm is more comfortable than blocking the upper arm, so blocking the forearm to measure FMD is advocated [27]. At 12 weeks, the damage of endothelium-dependent relaxation and endothelium-independent relaxation was further aggravated, which was closely related to pathological results. Liu et al. [28] used color Doppler ultrasound to measure the inner diameter changes of the brachial artery in healthy subjects under different conditions such as reactive congestion and intra-arterial injection of Ach and sodium nitroprusside and remeasured the inner diameter changes after administration of NG-monomethyl-L-arginine (LNMMA), a NO-dependent vasodilation response caused by Ach and reactive congestion. Endothelial-derived diastolic function was also greatly improved compared with the control group, and the transplanted endothelial progenitor cells did not affect the contractile function of arterial smooth muscle cells in injured vascular segments.

RETRACTED

In this study, we found that HAVEN's neighbor gene S1PR1 and its transcription factors can participate in the expression regulation of HAVEN and participate in the inflammatory reaction of vascular endothelial cells by regulating the expression of Enos and vcam-L. The possible mechanism of AKT downstream has not been deeply discussed, and it has been reported that mTOR can change as a downstream molecule of AKT. And mTOR is the main signal pathway of autophagy. It is suggested that *Rosa multiflora* may reduce brain edema induced by acute hypobaric hypoxia by inhibiting the overexpression of AQP1 and AQP4 in rat brain tissue, thus playing a protective role in the brain. In this paper, we observed the endothelium-dependent and endothelium-independent relaxation functions of blood vessels in different stages of atherosclerosis and their corresponding pathological changes. We thought that the endothelium-dependent relaxation function was damaged in the early stage of atherosclerosis. Although there was no change in general and under a light microscope, there were ultrastructural changes, which was the morphological basis for the decrease of endothelium-dependent relaxation function. Noninvasive detection of vascular endothelial function by Doppler ultrasound has attracted increasing clinical attention because of its simplicity, being painless, good repeatability, being economic, and accuracy.

## 6. Conclusion

To sum up, vascular endothelium can show dysfunction before atherosclerosis changes. Vascular endothelial dysfunction participates and influences the complex pathophysiological process of atherosclerosis from different angles and stages. Endothelial dysfunction can predict the development and prognosis of lesions. Autophagy and noncoding RNA play an important role in the occurrence, progression, and protection of cardiovascular diseases. The study of using miRNA agonists and antagonist mimetics provides hope for potential clinical application. Noninvasive detection of vascular endothelial function by Doppler ultrasound has attracted increasing clinical attention because of its simplicity, being painless, good repeatability, being economic, and accuracy.

RETRACTED

Although this method is simple and feasible, some problems need to be further improved. For example, the probe frequency of the ultrasonic diagnostic instrument used in this experiment is not high, which affects the image resolution. It is expected that higher frequency ultrasound can be applied to detect endothelial function in the future, and a more accurate conclusion can be drawn.

## Figures and Tables

**Figure 1:** EPC growth chart. (a) The first day of growth; (b) the second day of growth; (c) the third day of growth; (d) the 7th day of growth.

**Figure 2:** Changes of EPC proliferation curve.

**Figure 3:** Effect of autophagy on proliferation of EPCs.

**Figure 4:** NO content in plasma of rats in each group.

**Figure 5:** Changes of brain water content of rats in each group.

**Figure 6:** HE staining (×400) ((a) hippocampus; (b) cerebral cortex).

**Figure 7:** HAEC was transfected with siSIPRl and siLF2, respectively, and the expression of HAVEN was detected.

**Table 1:** Endothelium-dependent relaxation function of external iliac artery of rats in each group competes for endothelium-independent relaxation function.

Group	*n*	Endothelium-dependent vasodilation function	Independent relaxation function of vascular endothelium
Control group	6	15.36 ± 2.51	10.29 ± 2.71
Atherosclerosis model for 4 weeks	5	8.74 ± 1.05	9.96 ± 2.71
Atherosclerosis model in group A for 8 weeks	5	4.36 ± 0.88	6.68 ± 1.37
Group B: atherosclerosis model 12-week group	5	115 ± 0.49	4.88 ± 0.71

## Data Availability

Some or all data, models, or code generated or used during the study are available from the corresponding author by request.
